The article "Myopia in Chinese Adolescents: Its Influencing Factors and Correlation with Physical Activities" was retracted in 2023. Reasons: unreliable results or conclusions; concerns about the data; concerns about the peer review; concerns about the citations.

# Myopia in Chinese Adolescents: Its Influencing Factors and Correlation with Physical Activities

**DOI:** 10.1155/2022/4700325

**Published:** 2022-08-24

**Authors:** Yao Yin, Cheng Qiu, Yufei Qi

**Affiliations:** ^1^Beijing College of Finance and Commerce, No. 15, Shuuizi East Rd., Chaoyang District, Beijing, China; ^2^People's Public Security University of China, Huangyi Rd., Daxing District, Beijing, China; ^3^Central South University, 932 Lushan South Rd., Changsha, China

## Abstract

**Purpose:**

The study is conducted to analyze the risk factors and the protective factors of myopia in Chinese adolescents and its correlation with physical activities and then to provide 2 formulas to predict the probability of becoming myopic and the probability of preventing myopia.

**Methods:**

This is a cross-sectional study in which a questionnaire survey was conducted among 650 students aged 14-17 from 5 schools in Beijing in 2021. The students were divided into two groups: nonmyopia group and myopia group. Statistically significant variables were selected after the univariate analysis for a binary logistic regression analysis.

**Results:**

In the univariate analysis, 18 risk factors of myopia were found and 14 physical-activity-related protective factors were found. In the multivariate analysis, 5 independent factors were found to be positively related to myopia and could be used for calculating the probability of becoming myopic. The 5 factors are gender, staying up late playing smartphones, parental myopia, daily time spent on digital devices, and regular eye examinations. Five physical-activity-related factors were found to be positively related to the prevention of myopia and can be used for the calculation of the probability of preventing myopia. The 5 factors are regular physical activities, attitude towards physical education, daily time spent on in-school physical activities, daily time spent on after-school physical activities, and eye exercises.

**Conclusions:**

The influencing factors of myopia in adolescents mainly include heredity, habits of using eyes, and environment. Physical activities can effectively reduce the probability of becoming myopic in adolescents and promote eye health. Therefore, taking part in physical activities is an effective way to reduce the prevalence of myopia in adolescents.

## 1. Introduction

Eye health was defined by the Lancet Global Health Commission as maximized vision, ocular health, and functional ability, thereby contributing to overall health and well-being, social inclusion, and quality of life [1]. The International Agency for the Prevention of Blindness (IAPB) stressed in *2030 IN SIGHT* that the eye health of children and adolescents was the focus of future work and should be integrated into school health policy resulting in schools the world over routinely offering sight tests and eye health promotion and prevention information should be taught within education settings [2].

The article "Myopia in Chinese Adolescents: Its Influencing Factors and Correlation with Physical Activities" was retracted in 2023. Reasons: unreliable results or conclusions; concerns about the data; concerns about the peer review; concerns about the citations.

The incidence of myopia in China has increased significantly in recent years. Some pointed out that 20% to 50% of the students in primary school, 35% to 60% of the students in middle school, and 50% to 75% of the students in college are myopic in China in 2018 [3]. As of October 2021, 52.7% of the children and adolescents in China were myopic, and the rate was 2.5% higher than that in 2019 [4]. Schools, where children and adolescents carry out daily activities, are the main places for the improvement of their physical and mental health. The Ministry of Education attaches great importance to the prevention and control of myopia in young students and has formulated a specific work plan for it in 2018. Multiple measures and much effort have been taken to curb the prevalence of myopia.

Previous studies show that gender, age, region of habitation, family history of myopia, daily reading time, breaks while studying, daily time spent on digital devices, and learning piano are independent risk factors of myopia in primary school students in China [5]. The pathogenesis of myopia remains unclear so far, which may be related to genetic, environmental, and other factors. Some argued that the influence of environmental factors, such as bad habits of using eyes and visual fatigue, was greater than that of genetic factors [6, 7]. In summary, the eye health of children and adolescents is closely related to the environment, heredity, and intense use of the eyes.

It is regarded as an important part of student management, education, and teaching in China's School Management Standards for Compulsory Education that schools should help students to develop strong constitutions and reduce the prevalence of myopia among students. *Mingmu Gong*, a kind of Chinese eyesight improvement exercise, is said to have a significant effect on the recovery of students' eyesight, which helps to relax the eye muscles and accelerate the eye blood flow and further promote the recovery of eye vision [8]. Smartphone users are more likely to be myopic, showing a moderate positive correlation between playing smartphones and myopia. Outdoor activities reduce the probability of myopia, showing a strongly negative correlation between outdoor activities and myopia [9]. Compared with nonmyopic children, myopic children spend more time watching screens and shorter time on outdoor activities [10]. Outdoor activities help to prevent adolescents from being sedentary and improve their eyesight. Physical education should be integrated with the health service system to promote eye health education.

The article "Myopia in Chinese Adolescents: Its Influencing Factors and Correlation with Physical Activities" was retracted in 2023. Reasons: unreliable results or conclusions; concerns about the data; concerns about the peer review; concerns about the citations.

Based on an in-depth literature review, this study analyzed the influencing factors of myopia in adolescents and predicted the probability of becoming myopic through the analysis of the risk factors of myopia. Physical activities were important factors affecting eye health, and in this study, they were analyzed and used to predict the probability of preventing myopia.

## 2. Research Objects and Methods

### 2.1. Participants

A total of 650 questionnaires were distributed to 650 middle school students in Beijing using stratified sampling, and 610 of them were collected. After excluding 31 invalid questionnaires, there were 579 (89%) valid questionnaires left.

### 2.2. Research Variables

Based on previous studies, this study summarized the influencing factors of myopia in adolescents and the physical-activity-related factors, according to which the questionnaire was designed. 17 binary variables were investigated, such as gender, only child, playing video games, parental myopia, reading posture, writing posture, staying up late playing smartphones, and regular physical exercises. 21 continuous variables were investigated, such as diopter, daily time spent on digital devices, daily sleep duration, distance to the TV screen, illumination while studying, drinking milk, bedtime, get-up time, afternoon nap duration, breaks while studying, reading extracurricular books, daily time spent in reading in extremely weak or strong light, picky about food, eating whole grains and vegetables, frequency of visual acuity tests, regular eye examinations, attitude towards physical education, daily time spent on in-school physical activities, after-school physical activities, and eye exercises.

### 2.3. Statistical Methods

The data were statistically analyzed by SPSS 26.0. The continuous variables were first tested for normality, and those that do not conform to the normal distribution were analyzed by nonparametric tests. Binary logistic regression was performed for the multivariate analysis, and GraphPad 9.0 was used to draw figures. All participants agreed to participate in the study.

### 2.4. Ethical Approval

This research was approved by the independent ethics committee of the Institute of Clinical Pharmacology, Central South University (registered number: ctxy-140003). All methods were carried out in accordance with relevant guidelines and regulations. This study was carried out in compliance with the ARRIVE guidelines. Informed consent was obtained from caregivers, and all information was kept strictly confidential.

The article "Myopia in Chinese Adolescents: Its Influencing Factors and Correlation with Physical Activities" was retracted in 2023. Reasons: unreliable results or conclusions; concerns about the data; concerns about the peer review; concerns about the citations.

## 3. Results and Analysis

### 3.1. Univariate Analysis

The chi-square test and the nonparametric two-sample test were performed for the univariate analysis of 24 independent variables. The results are as follows (see Table 1).

The results in Table 1 show factors such as gender, playing video games, parental myopia, reading posture, writing posture, staying up late playing smartphones, diopter, daily time spent on digital devices, daily sleep duration, distance to the TV screen, illumination while studying, daily time spent on homework, breaks while studying, reading extracurricular books, daily time spent in reading in extremely weak or strong light, eating whole grains and vegetables, visual acuity tests, and regular eye examinations were found significant (*P* < 0.05). These factors were kept for the multivariate analysis. Factors such as only child, daily sleep duration, drinking milk, get-up time, afternoon nap duration, and picky about food were found not significant, which means they are not the influencing factors of myopia in adolescents. The details are shown in Figure 1.

### 3.2. Univariate Analysis of Physical-Activity-Related Factors

The chi-square test and the nonparametric two-sample test were performed for the univariate analysis of 13 independent variables. The results are as follows (see Table 2).

The results in Table 2 show that the myopia rate of adolescents who often took part in physical activities is significantly lower than those who occasionally took physical exercise (*P* < 0.05). The myopia rate of adolescents who often participated in football, basketball, table tennis, track and field, swimming, tennis, badminton, volleyball, dance, and other sports is low (*P* < 0.05). Continuous variables such as attitude towards physical education, daily time spent on in-school physical activities, after-school physical activities, and eye exercises were found significant, and they were kept for the multivariate analysis. The details are shown in Figure 2.

### 3.3. Multivariate Analysis of Influencing Factors of Myopia

18 significant factors were kept for the multivariate analysis using binary logistic regression, and the factors are gender, playing video games, staying up late playing smartphones, parental myopia, reading posture, writing posture, diopter, daily time spent on digital devices, distance to the TV screen, illumination while studying, bedtime, daily time spent on homework, breaks while studying, reading extracurricular books, daily time spent in reading in extremely weak or strong light, visual acuity tests, regular eye examinations, and eat whole grains and vegetables. The results are as follows in Table 3.

The article "Myopia in Chinese Adolescents: Its Influencing Factors and Correlation with Physical Activities" was retracted in 2023. Reasons: unreliable results or conclusions; concerns about the data; concerns about the peer review; concerns about the citations.

From the above analysis, it can be clearly concluded that gender is an independent factor affecting the incidence of myopia (*P* < 0.05), and the incidence of myopia in females is 1.679 times higher than that in males. Staying up late playing smartphones is an independent factor of myopia (*P* < 0.01), and the incidence of myopia in those spending a long time playing smartphones is 1.964 times higher than in those spending a short time staying up late playing smartphones. Parental myopia is an independent factor affecting the incidence of myopia (*P* < 0.01), and the incidence of myopia in those who have myopic parents is 1.880 times higher than in those who do not. Daily time spent on digital devices is an independent factor of myopia (*P* < 0.01), and the incidence of myopia in those spending a long time on digital devices is 1.721 times higher than that in those spending a short time on digital devices. Regular eye examinations is an independent factor affecting the incidence of myopia (*P* < 0.01), and the incidence of myopia in those who never (or rarely) have their eyes examined is 1.614 times higher than that in those who have regular eye examinations annually. The rest factors are not independent influencing factors of myopia (*P* > 0.05). From the above analysis, the forest plot of the five independent influencing factors of myopia was given.

Based on the above five factors in Figure 3 that significantly affect the incidence of myopia, a formula for predicting the probability of becoming myopic is given.

*Z* = −3.953 + 0.518∗1 (if gender = female) + 0∗1 (if gender = male) + 0.675∗1 (if staying up late playing smartphones = true) + 0∗1 (if staying up late playing smartphones = false) + 0.631∗1 (if parental myopia = true) + 0∗1 (if parental myopia = false) + 0.543∗3 (daily time spent on digital devices > 4 h) + 0.478∗2 (regular eye examinations = false).

(1) $$\begin{array}{c} P_{\text{myopia}}=\frac{1}{1+e^{-Z}}. \end{array}$$

The following is an example that shows how to predict the probability of becoming myopic of a female student who often stays up late playing smartphones, has myopic parents, spends more than 4 hours on digital devices every day, and rarely has her eyes examined.

(2) $$\begin{array}{c} Z=-3.953+0.518*1+0.675*1+0.631*1+0.543*4+0.478*2=0.999,\\ P_{\text{myopia}}=\frac{1}{1+e^{-\text{Z}}}=\frac{1}{1+e^{0.999}}=73\%. \end{array}$$

The probability of becoming myopic of the student is 73% (>50%), which means the student will be myopic.

### 3.4. Multivariate Analysis of the Correlation between Physical Activities and Myopia

In the univariate analysis, 5 significant factors were kept for multivariate analysis using binary logistic regression, and the factors are regular physical activities, daily time spent on in-school physical activities, after-school physical activities, eye exercises, and attitude towards physical education. The results are as follows in Table 4.

The article "Myopia in Chinese Adolescents: Its Influencing Factors and Correlation with Physical Activities" was retracted in 2023. Reasons: unreliable results or conclusions; concerns about the data; concerns about the peer review; concerns about the citations.

From the above analysis, it can be clearly concluded that regular physical activities is an independent factor reducing the incidence of myopia (*P* < 0.01), and the incidence of myopia in those who had regular physical activities was 0.523 times lower. Daily time spent on in-school physical activities (*P* < 0.001), after-school physical activities (*P* < 0.05), eye exercises (*P* < 0.01), and attitude towards physical education (*P* < 0.01) were all independent factors reducing the occurrence of myopia. According to the above analysis, the forest plot of the five independent influencing factors against myopia was given.

Based on the 5 factors in Figure 4 that significantly prevent myopia, a formula for predicting preventing myopia prevalence is given.

*Z* = 1.986 − 0.648∗1 (if regular physical activities = true) − 0.560∗3 (if daily time spent on in‐school physical activities = 40‐60 minutes) + 0.192∗2 (if after‐schoolphysical activities = occasionally) − 0.366∗3 (if eye exercises = often) + 0.276∗4 (if  attitude  to  physical  education = very like).

(3) $$\begin{array}{c} P_{\text{nonmyopia}}=\frac{1}{1+e^{-Z}}. \end{array}$$

The following is an example that shows how to predict the probability of preventing myopia of a student who takes part in physical activities for 40-60 minutes every day, occasionally takes part in after-school physical activities, often do eye exercises, and like PE lessons very much.

(4) $$\begin{array}{c} Z=1.986-0.648*1-0.560*3+0.192*2-0.366*3+0.276*4=0.51,\\ P_{\text{nonmyopia}}=\frac{1}{1+e^{-Z}}=\frac{1}{1+e^{-0.552}}=51\%. \end{array}$$

The probability of the student not being myopic is 51%, which means the student will not be myopic.

## 4. Discussion

The univariate analysis showed that factors like playing video games, parental myopia, reading posture, writing posture, distance to the TV screen, daily time spent on homework, breaks while studying, reading extracurricular books, daily time spent in reading in extremely weak or strong light, eating whole grains and vegetables, visual acuity tests, and regular eye examinations are influencing factor for myopia, which is consistent with Luo's study [11]. Students who play digital devices for a long time every day might have eyestrain even keratitis [12]. The incidence of myopia in girls was higher than that in boys, which is consistent with the results of Wen's study [5]. The difference may be due to different environments. Girls like to be quiet and study harder, while boys prefer outdoor activities. Parental myopia, long daily reading time, and less outdoor activity time are the risk factors associated with the increased incidence of myopia [13].

The article "Myopia in Chinese Adolescents: Its Influencing Factors and Correlation with Physical Activities" was retracted in 2023. Reasons: unreliable results or conclusions; concerns about the data; concerns about the peer review; concerns about the citations.

With the popularity of electronic products, most adolescents are equipped with learning and game devices. They often spend 3-4 hours reading, writing, and doing homework without rest, and sometimes they even stay up until the wee hours of the morning, which increases the burden on their eyes. The muscles inside and outside the eyes get tense and cannot get a good rest, which might lead to eye muscle spasms. The multivariate analysis of the significant factors was conducted after the univariate analysis of myopia, and the significant factors obtained by multivariate analysis were regarded as the independent influencing factors of myopia. Through binary logistic regression analysis, it was found that gender, parental myopia, staying up late playing smartphones, daily time spent on digital devices, and regular eye examinations were the independent influencing factors of myopia. According to these independent factors affecting myopia, this study attempted to give a formula for predicting the probability of becoming myopic.

The results of the univariate analysis of the correlation between physical activities and myopia showed that the incidence of myopia was lower in those that took part in regular physical activities and actively participated in sports (basketball, volleyball, and football). Continuous variables such as daily time spent on in-school physical activities, after-school physical activities, eye exercises, and attitude towards physical education are also influencing factors of myopia. Outdoor activities and physical activities are beneficial to reduce the incidence of myopia. For adolescents, sports such as basketball, volleyball, and badminton can effectively reduce the risk of becoming myopic [14]. Factors such as more outdoor activities, exposure to natural light, and outdoor environment are protective for the eyes of adolescents [15–18]. Through binary logistic regression analysis, it is found that regular physical activities, daily time spent on in-school physical activities, after-school physical activities, eye exercises, and attitude towards physical education are the main influencing factors in the prevention of myopia. Based on these independent factors, the prediction formula for preventing myopia is given and the probability of nonmyopia can be calculated according to the specific conditions of the students.

Potential limitations of our study should be mentioned. First of all, it is difficult to investigate the change of myopia with time by a cross-sectional study, and a multilevel linear model should be adopted to obtain a causal explanation in the future. Secondly, compared with previous review studies, this study may only be a potential myopia control strategy, and in future surveys, the time of physical activities and its impact on myopia need to be better defined and quantified.

The article "Myopia in Chinese Adolescents: Its Influencing Factors and Correlation with Physical Activities" was retracted in 2023. Reasons: unreliable results or conclusions; concerns about the data; concerns about the peer review; concerns about the citations.

## 5. Conclusions

(1) The results of the univariate analysis showed the influencing factors of myopia in adolescents and the factors related to physical activities that affect the prevalence of myopia. (2) The results of the multivariate analysis showed the independent influencing factors of myopia in adolescents and the independent influencing factors related to physical activities that affect the prevalence of myopia. (3) The significant factors in multivariate analysis were used to provide 2 formulas to predict the probability of becoming myopic and the probability of preventing myopia.

## Figures and Tables

**Figure 1:** Univariate analysis of the influencing factors of myopia.

**Figure 2:** Analysis of the correlation between physical activities and myopia.

**Figure 3:** Forest plot of the five independent influencing factors of myopia.

**Figure 4:** Forest plot of the five independent influencing factors protecting against myopia.

**Table 1:** Analysis of influencing factors of myopia.

Parameter		Groups		Myopia rate	*X* ^2^/*Z*	*P*
		Nonmyopia group	Myopia group			
Gender	Male	115	190	62.3%	5.543	0.019
	Female	78	196	71.5%		
Only child	No	94	191	67.0%	0.031	0.860
	Yes	99	195	66.3%		
Playing video games	Occasionally	67	97	59.1%	5.823	0.016
	Often	126	289	69.6%		
Parental myopia	No	76	107	58.5%	8.090	0.004
	Yes	117	279	70.5%		
Reading posture	Poor	123	288	70.1%	7.396	0.007
	Good	70	98	58.3%		
Writing posture	Poor	116	272	70.1%	6.250	0.012
	Good	77	114	59.7%		
Staying up late playing smartphones	Occasionally	116	194	62.6%	5.013	0.025
	Often	77	192	71.4%		
Diopter #		2 (1~4)	3 (2~4)		-4.579	<0.001
<2.0		75	40	10.40%		
2.0-4.0		27	105	27.20%		
4.0-6.0		35	105	27.20%		
6.0-8.0		38	94	24.40%		
>8.0		18	42	10.90%		
Daily time spent on digital devices #		2 (1~3.5)	3 (2~4)		-4.369	<0.001
<1 h		73	39	10.10%		
1-2 h		29	113	29.30%		
3-4 h		43	123	31.90%		
>4 h		48	111	28.80%		
Daily sleep duration #		2 (2~3)	2 (2~2.25)		-1.366	0.172
<6 h		29	75	19.40%		
6-8 h		109	215	55.70%		
>8 h		55	96	24.90%		
Distance to TV screen #		3 (2~4)	3 (2~4)		-2.238	0.025
<1 m		28	89	23.10%		
2-3 m		35	72	18.70%		
3-4 m		48	84	21.80%		
4-5 m		40	73	18.90%		
>5 m		42	68	17.60%		
Illumination while studying #		4 (2~5)	3 (2~4)		-2.97	0.003
Reading lamp (white light)		29	92	23.80%		
Reading lamp (yellow light)		36	64	16.60%		
Pendant lamp (white light)		29	83	21.50%		
Pendant lamp (white light)		45	73	18.90%		
Natural light (sunlight)		54	74	19.20%		
Drinking milk #		3 (2~4)	3 (2~4)		-1.188	0.235
Never		5	13	3.40%		
Occasionally		61	118	30.60%		
Often		57	148	38.30%		
Every day		70	107	27.70%		
Bedtime #		2 (1~3)	1 (1~2)		-2.857	0.004
After 24:00		91	222	57.50%		
23:00-24:00		50	105	27.20%		
22:00-23:00		36	33	8.50%		
21:00-22:00		16	26	6.70%		
Get-up time #		2 (1~3)	2 (1~3)		-0.783	0.434
Before 5:00		57	116	30.10%		
5:00-6:00		51	115	29.80%		
6:00-7:00		67	129	33.40%		
After 7:00		18	26	6.70%		
Afternoon nap duration #		2 (1~2)	2 (1~3)		-0.693	0.488
No		84	178	46.10%		
<20 minutes		72	101	26.20%		
20-40 minutes		29	72	18.70%		
>40 minutes		6	28	7.30%		
Daily time spent on homework #		2 (2~3)	3 (2~3)		-4.201	<0.001
<40 minutes		43	39	10.10%		
40-80 minutes		74	135	35.00%		
>80 minutes		76	212	54.90%		
Breaks while studying #		2 (1~2)	2 (2~3)		-3.451	0.001
Often		60	76	19.70%		
Rarely		89	180	46.60%		
Never		44	130	33.70%		
Reading extracurricular books #		2 (1~2)	2 (1.75~3)		-3.547	<0.001
Dislike		67	96	24.90%		
Like		93	173	44.80%		
Very like		33	117	30.30%		
Daily time spent in reading in extremely weak or strong light #		2 (1~3)	2 (2~3)		-2.528	0.011
<20 minutes		49	66	17.10%		
20-40 minutes		81	161	41.70%		
40-80 minutes		63	159	41.20%		
Picky about food #		4 (3~5)	4 (3~5)		-0.585	0.559
Extremely		4	10	2.60%		
Quite		10	24	6.20%		
Moderate		45	84	21.80%		
Slightly		49	111	28.80%		
Not		85	157	40.70%		
Eating whole grains and vegetables #		2 (2~3)	3 (2~3)		-4.243	<0.001
Never		84	230	59.60%		
Rarely		68	120	31.10%		
Often		41	36	9.30%		
Visual acuity tests #		1 (1~2)	1 (1~2)		-2.011	0.044
Rarely		121	212	54.90%		
Once every 6 months		45	95	24.60%		
Once every 3 months		27	79	20.50%		
Regular eye examinations #		2 (1~2)	2 (1~2)		-2.800	0.005
Never		91	132	34.20%		
Rarely		80	199	51.60%		
Annually		22	55	14.20%		

^∗^Factors ending with # are not normally distributed according to the results of the SW normality test.

The article "Myopia in Chinese Adolescents: Its Influencing Factors and Correlation with Physical Activities" was retracted in 2023. Reasons: unreliable results or conclusions; concerns about the data; concerns about the peer review; concerns about the citations.

**Table 2:** Analysis of the correlation between physical activity and myopia.

Parameter		Groups		Myopia rate	*X* ^2^/*Z*	*P*
		Nonmyopia group	Myopia group			
Regular physical activities	No	109	272	71.40%	11.190	0.001
	Yes	84	114	57.60%		
Football	Rarely	135	299	68.90%	3.869	0.049
	Occasionally	58	87	60.00%		
Basketball	Rarely	79	194	71.10%	4.491	0.034
	Occasionally	114	192	62.70%		
Ping pang	Rarely	112	283	71.60%	13.866	<0.001
	Occasionally	81	103	56.00%		
Track and field	Rarely	75	186	71.30%	4.520	0.033
	Occasionally	118	200	62.90%		
Swimming	Rarely	112	271	70.80%	8.519	0.004
	Occasionally	81	115	58.70%		
Tennis	Rarely	127	285	69.17%	4.044	0.044
	Occasionally	66	101	60.48%		
Badminton	Rarely	82	206	71.50%	6.093	0.014
	Occasionally	111	180	61.90%		
Volleyball	Rarely	68	180	72.58%	6.828	0.009
	Occasionally	125	206	62.24%		
Dance	Rarely	54	143	72.60%	4.713	0.030
	Occasionally	139	243	63.60%		
Attitude to physical education #		4 (3~4)	3 (3~4)		-3.284	0.001
Negative		96	134	34.70%		
Indifferent		27	64	16.60%		
Positive		58	157	40.70%		
Very positive		12	31	8.00%		
Daily time spent on in-school physical activities #		2 (1~3.5)	3 (2~4)		-5.074	<0.001
<20 minutes		48	111	28.80%		
20-40 minutes		29	113	29.30%		
40-60 minutes		43	123	31.90%		
>60 minutes		73	39	10.10%		
After-school physical activities #		3 (2~4)	3 (2~4)		-2.209	0.027
Rarely		72	116	30.10%		
Occasionally		46	92	23.80%		
Sometimes		61	127	32.90%		
Often		14	51	13.20%		
Eye exercises #		2 (1~3)	1 (1~2)		-3.453	0.001
Never		84	217	56.20%		
Rarely		51	107	27.70%		
Occasionally		42	36	9.30%		
Often		16	26	6.70%		

^∗^Factors ending with # are not normally distributed according to the results of the SW normality test.

**Table 3:** Binary logistic analysis of influencing factors of myopia.

Parameter	*B*	S.E.	Wald	DF	*P*	OR	OR 95% CI	
							Minimum	Maximum
Gender	0.518	0.206	6.302	1	0.012	1.679	1.120	2.516
Playing video games	0.006	0.761	0.000	1	0.993	1.006	0.226	4.474
Staying up late playing smartphones	0.675	0.232	8.488	1	0.004	1.964	1.247	3.093
Parental myopia	0.631	0.216	8.507	1	0.004	1.880	1.230	2.872
Reading posture	-0.590	0.763	0.598	1	0.439	0.555	0.124	2.472
Writing posture	-0.365	0.21	3.034	1	0.082	0.694	0.460	1.047
Diopter	0.136	0.166	0.676	1	0.411	1.146	0.828	1.587
Daily time spent on digital devices	0.543	0.203	7.164	1	0.007	1.721	1.156	2.561
Distance to TV screen	-0.072	0.075	0.905	1	0.341	0.931	0.803	1.079
Illumination while studying	-0.116	0.080	2.100	1	0.147	0.890	0.760	1.042
Bedtime	-0.167	0.115	2.095	1	0.148	0.847	0.676	1.061
Daily time spent on homework	0.130	0.307	0.179	1	0.673	1.139	0.623	2.080
Breaks while studying	0.066	0.212	0.098	1	0.754	1.069	0.706	1.618
Reading extracurricular books	0.081	0.208	0.153	1	0.696	1.085	0.721	1.631
Daily time spent in reading in extremely weak or strong light	0.221	0.147	2.273	1	0.132	1.247	0.936	1.663
Visual acuity tests	0.168	0.134	1.581	1	0.209	1.183	0.910	1.537
Regular eye examinations	0.478	0.153	9.723	1	0.002	1.614	1.194	2.180
Eating whole grains and vegetables	-0.390	0.310	1.581	1	0.209	0.677	0.369	1.243
Constants	-2.393	1.534	2.433	1	0.119	0.091		

**Table 4:** Binary logistic analysis of the correlation between physical activities and myopia.

Parameter	*B*	S.E.	Wald	DF	*P*	OR	OR 95% CI	
							Minimum	Maximum
Regular physical activities	-0.648	0.196	10.965	1	0.001	0.523	0.357	0.768
Daily time spent on in-school physical activities	-0.560	0.092	37.376	1	<0.001	0.571	0.477	0.684
After-school physical activities	0.192	0.094	4.177	1	0.041	1.211	1.008	1.456
Eye exercises	-0.366	0.102	13.002	1	0.000	0.693	0.568	0.846
Attitude towards physical education	0.276	0.094	8.570	1	0.003	1.317	1.095	1.584
Constants	1.986	0.453	19.26	1	<0.001	7.287		

The article "Myopia in Chinese Adolescents: Its Influencing Factors and Correlation with Physical Activities" was retracted in 2023. Reasons: unreliable results or conclusions; concerns about the data; concerns about the peer review; concerns about the citations.

## Data Availability

The datasets generated during and/or analyzed during the current study are available from the corresponding author on reasonable request.
